The article "Retrospection of Nonlinear Adaptive Algorithm-Based Intelligent Plane Image Interaction System" was published in 2022. Journal: Comput Intell Neurosci.

# Retrospection of Nonlinear Adaptive Algorithm-Based Intelligent Plane Image Interaction System

**DOI:** 10.1155/2022/3502830

**Published:** 2022-03-09

**Authors:** Zixi Guan, Raja Varma Pamba, Bhuvaneswari Balachander, Deepak Kumar Khare, Nabamita Deb, Rajasekhar Boddu

**Affiliations:** ^1^Shenyang City University, School of Film and Television Media, Liaoning, Shenyang 110112, China; ^2^LBS Institute of Technology for Women, Poojapura, Thiruvanathapuram, Kerala, India; ^3^Saveetha School of Engineering, Saveetha Institute of Medical and Technical Sciences, Chennai, Tamil Nadu, India; ^4^Department of Information Technology, Institute of Engineering and Technology, Dr. Rammanohar Lohiya Avadh University, Ayodhya, UP, India; ^5^Department of Information Technology, Gauhati University, Assam 781014, India; ^6^Department of Software Engineering, College of Computing and Informatics, Haramaya University, Dire Dawa, Ethiopia

## Abstract

This paper introduces the application and classification of an adaptive filtering algorithm in the image enhancement algorithm. And the filtering noise reduction impact is compared using MATLAB software for programming, image processing, LMS algorithm, RLS algorithm, histogram equalisation algorithm, and Wiener filtering method filtering noise reduction effect. To optimize the intelligent graphic image interaction system, the proposed nonlinear adaptive algorithm of intelligent graphic image interaction system research is based on the digital filter and adaptive filtering algorithm for simulation experiment. The experimental results of several noise index data filtering algorithms show that the fuzzy coefficient *k* of LMS index is 0.86, RLS index is 0.91, the histogram equalization index is 0.53, and the Wiener filtering index is 0.62. LMS index of quality index *Q* is 0.90, RLS index is 0.95, histogram equalization index is 0.58, Wiener filtering index is 0.65. According to the above results, comparing LMS with the RLS method and according to SNR, *k*, and *Q* values in the simulation results in the process of processing, it is found that the convergence speed of the RLS algorithm is obviously better than that of the LMS algorithm, and the stability is also good. Additionally, the differential imaging data can provide a strong reference for the clinical diagnosis and qualitative differentiation of TBP and CP, and MSCT is worthy of extensive application in the clinical diagnosis of peritonitis. The processing effect of the image with high similarity to the original image is greatly improved compared with the histogram equalization and Wiener filtering methods used in the simulation.

## 1. Introduction

Rapid breakthroughs in scientific knowledge have created a vast amount of picture data in a variety of industries, including entertainment, art galleries, fashion design, education, medical, and industry. We frequently need to efficiently store and retrieve visual data in order to complete given jobs and make decisions. As a result, establishing appropriate tools for picture retrieval from big image libraries is difficult. In picture retrieval, two methodologies are often used: text-based methodology and content-based methodology. The photos in the text-based system are manually labeled with text descriptors before being employed by a database management system to do image retrieval [1, 2]. With the progress of science and technology and the development of social productivity, the control objects in the actual industrial process are more and more complex, and there are many strong nonlinearity, uncertainty, and time variations, so people's requirements for the control of the actual production process are increasingly accurate. Therefore, the classical linear feedback control has been difficult to adapt to the needs [3]. The nonlinear system is approximately linearized through the transformation of input and state variables. Although it is convenient for people to understand the characteristics of the system more conveniently and simply, it is difficult to describe the nonlinear characteristics of the original system, and the linearized system cannot well reflect the nonlinear characteristics of the actual system [4]. The nonlinear control theory, in the late twentieth century based on the original control theory, became the dominant trend in the 21^th^ century. Adaptive control theory has gained importance as a subset of nonlinear control theory and has become a research priority [5]. When the parameters of the controlled system are uncertain or vary little, the traditional adaptive control shows good control effect. It is based on the input and output of the control system and the online identification of system parameters. In the process of control, a more accurate model of the system is gradually obtained, and the design of the controller is combined with the system identification. Because the model of the system gradually approximates the actual model, the interference caused by the uncertainty of the model is greatly reduced, and the utility of the designed controller is also getting better and better [6]. Conceptually, the controller is designed to be adaptable. The adaptive controller's advantages and disadvantages are determined by the controller's design method on the one hand and the system identification algorithm's calculation speed on the other. The algorithm converges quickly and has a good control effect if the chosen initial value is close to the real value. As a result, the adaptive controller assumes that the operating environment is either constant or slowly changing over time. The controller can then be built using either a model with constant parameters or one with slow changes. If the system parameters have a large jump, for example, in display industrial control, boundary condition changes, subsystem failure, external interference, and other problems often make the system jump from the original working point to the new working point, the transient error at the jump time is often very large and the convergence rate of identification algorithm is reduced. The control effect is greatly reduced, so another new control method is needed [7]. To better solve the previous problems, a multimodel adaptive control method can be adopted to control the controlled system. An and Liu proposed an algorithm for a specific quadratic index and obtained the corresponding explicit feedback control law. The theory of the nonlinear control system method mainly includes Lyapunov method synthesis of asymptotically stable system, variable structure control, global linearization, and regularization [8]. Comprehensive surveys exist on content-based image retrieval (CBIR) [9]. CBIR is a technique that helps to organize digital image archives based on their visual content. CBIR covers anything from an image similarity tool to a comprehensive image annotation engine, according to this definition. CBIR's classification as a field of research places it in an unusual position within the scientific world. We see people from various fields, such as computer vision, human-computer interaction, database systems, information retrieval, machine learning, web and data mining, information theory, statistics, and psychology, contributing and becoming part of the CBIR community. Surveys also exist on closely related topics such as relevance feedback [10], applications to art and cultural imaging [11], and face recognition [12].

The article "Retrospection of Nonlinear Adaptive Algorithm-Based Intelligent Plane Image Interaction System" was published in 2022. Journal: Comput Intell Neurosci.

Liu found defects in their existing theories, which are actually universal in nonlinear systems. The defects are mainly reflected in two aspects: the reversible problem of the nonlinear system and the structural problem under dynamic feedback. Both have long been the focus and difficulty of research. The problem of the nonlinear system has not been clearly understood, and the design of dynamic feedback is also stuck in the initial stage [6]. Liu et al. used a linear algebra method to study the structural characteristics of nonlinear systems from a new perspective [7]. Therefore, in this case, the control of nonlinear systems has a completely new development. On the basis of the current research, this paper mainly introduces the application and classification of the adaptive filtering algorithm in the image enhancement algorithm and uses MATLAB software for programming and image processing. The LMS algorithm, RLS algorithm, histogram equalization algorithm and Wiener filtering method filtering noise reduction effect is compared. According to the experimental results of the noise reduction index data of several filtering algorithms, the LMS index of fuzzy coefficient *k* is 0.86, the RLS index is 0.91, the histogram equilibrium index is 0.53, and the Wiener filtering index is 0.62. The LMS index of quality index *Q* is 0.90, RLS index is 0.95, histogram equalization index is 0.58, Wiener filtering index is 0.65. It is proved that the processing effect of the image with high similarity to the original image is greatly improved compared with the histogram equalization and Wiener filtering methods used in the simulation in this paper. Comparing LMS with the RLS method, according to SNR, *k*, and *Q* values in the simulation results, it can be seen that both methods have better image processing effects, among which RLS is better. Moreover, in the process of processing, it is found that the convergence speed of the RLS algorithm is obviously better than that of the LMS algorithm, and the stability is also good [13].

## 2. Method

### 2.1. Concept of Adaptive Filtering

Adaptive filters are commonly employed in image processing to enhance or restore data by decreasing noise without significantly distorting the image's features. The literature on adaptive filtering is vast, and it is difficult to cover it all in a single chapter. However, much of the study has been concentrated on one-dimensional (1D) signals. Such techniques are not immediately applicable to image processing, and there are no easy ways to extend 1D technique to higher dimensions, owing to the fact that data points in dimensions more than one do not have a unique ordering. Because higher-dimensional medical imaging data are common, we choose to focus this study on adaptive filtering techniques that can be applied to multiple signals (2D pictures, 3D volumes, and 4D time volumes) [14, 15]. Adaptive filtering methods mainly include digital filters and adaptive algorithms. There are two kinds of digital filters commonly used for adaptive filtering; one is FIR (two-dimensional finite impulse response) digital filter; the other is IIR (two-dimensional infinite impulse response) digital filter. The commonly used adaptive filtering algorithms mainly include the following categories: least mean square algorithm (LMS), recursive least square algorithm (RLS), adaptive filtering algorithm based on neural network, adaptive filtering algorithm based on QR decomposition, adaptive filtering algorithm based on the unified model, and adaptive algorithm based on high order simulant. Among them, the LMS algorithm is divided into two types: variable step size algorithm and transform domain algorithm. Due to its wide applicability, the adaptive filtering algorithm has been applied in many fields such as image enhancement and echo cancellation [16]. When passed through a nonlinear function, for any nonlinear function, UKF is the Gaussian filters such that the posterior mean and covariance can be accurate to the second order, but EKF can only obtain the accuracy of the first order. Moreover, the calculation of mean and variance only involves standard vector and matrix operations, which makes the algorithm of UKF suitable for any dynamic model. At the same time, because there is no need to calculate the Jacobian matrix of the nonlinear function, the UKF algorithm is faster than EKF. However, UKF still approximates the posterior probability density of the system state by Gaussian distribution, so in the case of non-Gaussian PDF of the system state, the filtering result will have a great error. The study of nonlinear control theory and linear control theory is almost simultaneous. However, due to the complexity and diversity of the nonlinear system, each part of the system influences each other and produces the equilibrium. Until now, it has not been accurately described and understood. For example, there are many kinds of stability that describe the zero point of a nonlinear system. Any singular equilibrium point leads to a more complex convergence of the system. In addition, there is no good mathematical description tool for nonlinear control systems. Therefore, linear control methods still occupy the main position in practical application, and most nonlinear control theories need to be developed.

The article "Retrospection of Nonlinear Adaptive Algorithm-Based Intelligent Plane Image Interaction System" was published in 2022. Journal: Comput Intell Neurosci.

### 2.2. Adaptive Filter and Digital Filter

Two-dimensional finite impulse response digital filter, also known as an FIR digital filter, is a kind of digital filters, which is more commonly seen in two-dimensional digital signal processing, in the application of adaptive filtering in image processing. Given that medical images are mostly two-dimensional gray images and FIR digital filters have a certain length in both dimensions, a stable filtering function can be achieved. The extended Kalman filter (EKF) is a classical method to deal with nonlinear systems [17]. The idea of EKF is to linearize the nonlinear vector functions *φ* and H of the stochastic nonlinear system model to get the linearized system model and then apply the basic equation of Kalman filter to solve the nonlinear filtering problem. The EKF algorithm is simple and easy to implement. It is one of the most commonly used nonlinear filtering methods. However, due to the linearization processing method of Taylor expansion, the filtering result of EKF can be close to the true value only when the state equation and observation equation of the system are close to linear and continuous [18]. When the state equation and observation equation are seriously nonlinear, the filtering result of EKF will be very bad. The filtering results of EKF are also related to the statistical characteristics of state noise and observation noise. In the recursive filtering process of EKF, the covariance matrix of state noise and observation noise remains unchanged. If the estimation of the two noise covariance matrices is not accurate enough, it is easy to produce error accumulation, leading to the divergence of filtering. Another disadvantage is that it is not easy to determine the initial state, which causes the state estimation accuracy to be sometimes low in application, and the divergence of filtering is easy to occur [19].

In this paper, the digital filter adopts the FIR digital filter. In the design process, the size of the two-dimensional matrix is set as *N*_1_ × *N*_2_, and the order of the two dimensions is *N*_1_ − 1, *N*_2_ − 1, respectively. The frequency response function of the filter is shown in the formula as follows:

(1) $$\begin{array}{c} H\left(e^{j\omega_{1}},e^{j\omega_{2}}\right)=\sum_{n_{2}=0}^{N_{2}-1}\sum_{n_{1}=0}^{N_{1}-1}h_{d}\left(n_{1},n_{2}\right)e^{-j\left(n_{1}\omega_{1}+n_{2}\omega_{2}\right)}. \end{array}$$

Here, *ω*_1_, *ω*_2_ is the frequency of the two dimensions, and its value range is [−*π*, *π*].

### 2.3. Adaptive Filtering Algorithm

An adaptive algorithm is one that adjusts its behaviour as it runs, based on the information available and a reward structure that has been designed in advance (or criterion). The tale of recently received data, information on available computational capabilities, or other run-time acquired (or a priori known) knowledge about the environment in which it operates are examples of such information. The adaptive filtering algorithm mainly includes the LMS method and the RLS method. In this paper, in the process of research on the adaptive filtering algorithm, first of all, the governing equation of two kinds of adaptive filtering algorithm is analyzed and deduced, and the two algorithms are simulated by the programming software MATLAB, and the effect of the two algorithms in the actual application process is compared:

(1) LMS method is a least mean square algorithm; the algorithm of time early is developed on the basis of the Wiener filtering method; with Wiener filtering solution as the initial value, by using the steepest descent method as a recurrence formula and iterative calculation, the optimal solution is finally obtained, as shown in the formula as follows:.
  (2) $$\begin{array}{c} y\left(n\right)=W^{T}\left(n\right)X\left(n\right),\\ e\left(n\right)=d\left(n\right)-y\left(n\right),\\ W\left(n+1\right)=W\left(n\right)+2\mu X\left(n\right)e\left(n\right), \end{array}$$
where *X*(*n*) is the input reference vector value; *μ* represents the space (time) step factor of the weighted vector of the input signal after filtering; *y*(*n*) is the output value of the filter; *e*(*n*) is output simultaneously as the error signal; *W*(*n*) represents both the weighted vector of the digital signal of the input image and the coefficient vector of the filter itself, and *W*(*n*) is expressed in the formula as follows:
  (3) $$\begin{array}{c} W\left(n\right)={\left[b_{0}\left(n\right),b_{1}\left(n\right),\ldots ,b_{n-1}\left(n\right)\right]}^{T}, \end{array}$$
where N represents the length of the selected filter. During the calculation of the LMS algorithm, the following steps should be followed: initialization: determine the initial value of the image to be processed and determine *W*(0) at the initial time; iteration calculation (iteration): iteration step *n*=0.1,…,; output *y*(*n*); estimate the calculation error: output *e*(*n*); update the input image signal: output *W*(*n*+1)=*W*(*n*)+2*μX*(*n*)*e*(*n*) in the process of the LMS algorithm design and calculation, attention should be paid to the setting of µ value, which has a great impact on the convergence and robustness of the algorithm. To ensure the stability of the iterative process, the value is generally selected as 0 < *μ* < 2MPin, and Pin is the input power in the calculation process. The adaptive algorithm process is shown in Figure 1.
(2) RLS algorithm, namely, recursive least squares algorithm, is based on the LMS algorithm. The difference is that in the process of filtering, the calculation of mean square error takes the variable length image input signal as the object and adds the weighted factor that changes with time. Compared with the LMS method, the error representation in this algorithm is shown in the formula as follows:

(4) $$\begin{array}{c} \xi \left(k\right)=\sum_{n=1}^{k}\theta \left(k,n\right){\left|\varepsilon \left(n\right)\right|}^{2}, \end{array}$$

where *n* = 1, 2,…, *k* in the above equation; *θ*(*k*, *n*) is the added weighting factor 0 ≤ *θ* ≤ 1 that changes with time.

The article "Retrospection of Nonlinear Adaptive Algorithm-Based Intelligent Plane Image Interaction System" was published in 2022. Journal: Comput Intell Neurosci.

In the above equation, *a*⟶1^−^ sorted the two equations to obtain the mean square error equation of the RLS algorithm, as shown in the following formula:.

(5) $$\begin{array}{c} \zeta \left(k\right)=\sum_{n=1}^{k}a^{k-n}\cdot {\left|\varepsilon \left(n\right)\right|}^{2}. \end{array}$$

In the calculation process of the RLS algorithm, when *ζ*(*k*) obtains the minimum value, it can be understood that the following equivalence relationship exists, as shown in the following formula:

(6) $$\begin{array}{c} R\left(k\right)\cdot \omega^{*}\left(k\right)=p\left(k\right). \end{array}$$

In this formula, the first term on the left side and the term on the right side of the equation are defined as follows:

(7) $$\begin{array}{c} R\left(k\right)=\sum_{n=1}^{k}a^{k-n}\cdot x\left(n\right)\cdot x^{H}\left(n\right),\\ p\left(k\right)=\sum_{n=1}^{k}a^{k-n}\cdot x\left(n\right)\cdot d^{H}\left(n\right). \end{array}$$

The weight coefficient *ω*^*∗*^(*k*) is the minimum value of *ζ*(*k*), and the calculation formula of *ω*^*∗*^(*k*) is derived; that is, the calculation of the weight vector is shown as follows:

(8) $$\begin{array}{c} \omega \left(k\right)=\omega \left(k-1\right)+r\left(k\right)\cdot \eta \left(k\right), \end{array}$$

where some orthogonal vector *η*(*k*)=*d*(*k*) − *ω*^*H*^(*k* − 1) · *x*(*k*), *d*(*k*) is determined; *r*(*k*) is the value in the inverse of the target matrix *Q*(*k*).

## 3. Results and Analysis

In this paper, MATLAB software is used to program the above two algorithms, which are used to process the image in this paper. The processing method is as follows: firstly, the original image (510 × 400 × 3) is processed with noise, and Gaussian noise (*E* = 0.25) is added to the original image. Then, the algorithm designed in this paper is used to process the image and compared with the histogram equalizer and Wiener filtering methods. The software implementation process is shown in Figure 2. An adaptive filter is a system with a linear filter and a transfer function controlled by variable parameters that may be adjusted using an optimization technique. Almost all adaptive filters are electronic filters due to the complicated of the optimization techniques. For some applications, adaptive filters are required because some variables of the required production process (for example, the positions of reflected surfaces in a reverberant space) are unknown or changeable. The closed loop adaptive filter streamlines its transfer function with feedback in the form of an error signal.

The time domain of its input signal is shown in Figure 3. Time domain analysis is particularly useful for circuit designs with antennas where a designer may encounter stray signals and reflections. Time domain signal processing enables an engineer to separate extraneous signals in time from the desired signal, thereby identifying the contaminated signals.

The article "Retrospection of Nonlinear Adaptive Algorithm-Based Intelligent Plane Image Interaction System" was published in 2022. Journal: Comput Intell Neurosci.

The mathematical form of SNR is PSNR, and at PSNR = 10, 1*g*(255^2^/*MSE*), where MSE is the root mean square value of the corresponding point before and after filtering,

(9) $$\begin{array}{c} MSE=\frac{1}{WH}\sum_{i=1}^{WH}{\left(x_{i}-{\bar{x}}_{i}\right)}^{2}. \end{array}$$

The larger the PSNR value is, the greater the proportion of the effective signal in the total signal is. The fuzzy coefficient mainly represents the comparison between the edge energy of the processed image and the original image, and its mathematical expression is shown as follows:

(10) $$\begin{array}{c} k=\frac{s_{i,out}}{s_{i,in}}. \end{array}$$

The closer the score on the right is to 1, the better the treatment quality is. The quality index *Q* is the most obvious index that represents the image processing effect. There is a big gap between the image processed by histogram equalization and the original image. Several methods in the simulation were quantitatively compared, with signal-to-noise ratio (SNR), fuzzy coefficient, and quality index as the main indicators. The comparison results are shown in Table 1.

## 4. Discussion

Based on the digital filter and adaptive filtering algorithm for the simulation and experimental results of several noise index data filtering algorithms, the fuzzy coefficient *k* of LMS index is 0.86, RLS index is 0.91, histogram equalization index is 0.53, and the Wiener filtering index is 0.62. LMS index of quality index *Q* is 0.90, RLS index is 0.95, histogram equalization index is 0.58, and Wiener filtering index is 0.65. According to the above results, comparing LMS with the RLS method and according to SNR, K, and Q values in the simulation results, it can be seen that both methods have better image processing effects, among which RLS is better. In the process of processing, it is found that the convergence speed of the RLS algorithm is obviously better than that of the LMS algorithm, and the stability is also good. Throughout this study, there were significant differences between patients with TBP and patients with CP in abdominal asitoneal fluid, parietal peritoneal changes, omentum changes, and mesentery changes, indicating that MSCT can achieve the acquisition of many image data related to pathological changes in patients with TBP and CP. The difference between the adaptive filtering algorithm and other filtering algorithms, such as Wiener filtering and Kalman filtering, lies in that the filtering coefficient of this algorithm is not fixed but changes correspondingly with the change of image signal and noise. Wiener filter and Kalman filter are the traditional simple linear filters, which have great limitations in image noise processing. In the adaptive filtering algorithm, the adaptive filter parameters determine its obvious advantages in image noise processing and image signal enhancement.

The article "Retrospection of Nonlinear Adaptive Algorithm-Based Intelligent Plane Image Interaction System" was published in 2022. Journal: Comput Intell Neurosci.

## 5. Conclusions

In the present work, based on the nonlinear adaptive algorithm that projected intelligent graphic image interaction system research and based on the digital filter and adaptive filtering algorithm for the simulation and experimental findings of different noise index data filtering algorithms, the fuzzy coefficient *k* of LMS index is 0.86, RLS index is 0.91, histogram equalization index is 0.53, and the Wiener filtering index is 0.62. The LMS index of quality index *Q* is 0.90, RLS index is 0.95, histogram equalization index is 0.58, and Wiener filtering index is 0.65. According to the above results, comparing LMS with the RLS method and according to SNR, K, and Q values in the simulation results, it can be seen that both methods have better image processing effects, among which RLS is better. In the process of processing, it is found that the convergence speed of the RLS algorithm is obviously better than that of the LMS algorithm, and the stability is also good. Throughout this study, there were significant differences between patients with TBP and patients with CP in abdominal asitoneal fluid, parietal peritoneal changes, omentum changes, and mesentery changes, indicating that MSCT can achieve the acquisition of many image data related to pathological changes in patients with TBP and CP. The adaptive filtering algorithm differs from other filtering algorithms such as Wiener and Kalman filtering in that the filtering coefficient of this algorithm is not set but evolves in response to changes in picture signal and noise. Traditional simple linear filters such as the Wiener and Kalman filters have significant limitations in image noise processing. The adaptive filtering algorithm's obvious advantages in image noise processing and image signal enhancement are ascertained by the adaptive filter parameters.

## Figures and Tables

**Figure 1:** Flowchart of adaptive algorithm.

**Figure 2:** Block diagram of software implementation of adaptive filter.

**Figure 3:** Time-domain diagram of input signal.

**Table 1:** Comparison of noise reduction indexes of several filtering algorithms.

Algorithm	LMS	RLS	Histogram equalization	Wiener filtering
SNR	40.5 dB	42.5 dB	21.2 dB	25.1 dB
Fuzzy system k	0.86	0.91	0.53	0.62
Quality index Q	0.90	0.95	0.58	0.65

## Data Availability

All the data used to support the findings of this study are included within the article.
